The article "Effect of Neutralizer on Transparency of Nucleating Agent-Containing Polypropylene" was published in 2021. Journal: Polymers (Basel).

# Effect of Neutralizer on Transparency of Nucleating Agent-Containing Polypropylene

**DOI:** 10.3390/polym13050680

**Published:** 2021-02-24

**Authors:** Shohei Iwasaki, Yohei Uchiyama, Miwa Tenma, Masayuki Yamaguchi

**Affiliations:** 1 School of Materials Science, Japan Advanced Institute of Science and Technology, 1-1 Asahidai, Nomi, Ishikawa 923-1292, Japan; s2020004@jaist.ac.jp (S.I.); mi.temma@teijin.co.jp (M.T.); 2 Research & Development Department, Research & Development Division, New Japan Chemical Co., Ltd., 13 Yoshijima, Yaguracho, Fushimi, Kyoto 612-8224, Japan; uchiyama-y@nj-chem.co.jp

**Keywords:** polypropylene, nucleating agent, neutralizer, transparency, dynamic mechanical properties

## Abstract

The effects of neutralizer species on the transparency of injection-molded plates were studied using isotactic polypropylene (PP) containing a crystal nucleating agent—i.e., 1,3:2,4-bis-*o*-(4-methylbenzylidene)-d-sorbitol (MDBS). A plate containing lithium stearate (StLi) was more transparent than one containing calcium stearate (StCa) when the MDBS content was 0.1 wt. %. The addition of StLi accelerated the formation of MDBS fibers and the crystallization of PP. However, when the MDBS content was 1.0 wt. %, StCa improved the transparency more effectively than StLi. These results indicate that the combination of an appropriate amount of MDBS and the correct neutralizer species is critical for enhancing the transparency of injection-molded PP plates.

## 1. Introduction

The demand for isotactic polypropylene (PP) with excellent transparency, especially in the form of injection-molded products, has been increasing in recent years. Industrially, the following methods are used to reduce light scattering: (1) the addition of nucleating agents [1,2,3], (2) copolymerization with ethylene or butene-1 [4,5,6], (3) rapid solidification [7,8], and (4) film stretching [9,10]. Specific nucleating agents known as clarifiers are often used in injection-molded products because they do not cause loss of rigidity [2,11,12,13,14]. Adding clarifiers does not require expensive equipment such as a biaxial stretching machine. Sorbitol derivatives are particularly popular clarifiers. Sorbitol-based nucleating agents melt in molten PP [15,16,17,18]. They appear as fibers with diameters of several nanometers owing to segregation/crystallization during the cooling process [13,19,20,21,22]. The fibers then act as nuclei for PP crystallization. Various attempts have been made to elucidate the mechanism by which sorbitol derivatives confer transparency on injection-molded products [23,24,25]. According to these studies, the addition of a sorbitol derivative greatly affects the structures of the skin and core layers of injection-molded products. In the skin layer, transcrystallization by the fibrous nucleating agents results in a high degree of molecular orientation in the flow direction [20,26,27,28,29]. Owing to the high level of molecular orientation, the correlation length—i.e., the size of the scattering units—exceeds the wavelength of visible light. This reduces the light scattering caused by anisotropic polarizability. In the core layer, spherulites—which generally occur in PP products in the absence of a nucleating agent—do not develop. This is because there are numerous nucleating sites on the fibers, which form a network structure. As a result, light scattering due to spherulites is reduced [30,31]. However, in the absence of a flow field in the core, the segregation/solidification of sorbitol derivatives often results in extensive agglomeration, leading to light scattering. Therefore, excess sorbitol derivatives often confer poor transparency [2,18,32,33,34,35].

The article "Effect of Neutralizer on Transparency of Nucleating Agent-Containing Polypropylene" was published in 2021. Journal: Polymers (Basel).

As explained, the formation of fibers by the sorbitol derivative in the molten PP is important for the transparency of the injection-molded product [25,32,36,37,38,39], which can be modified by another polar compound [40,41]. Therefore, the present study focused on the effect of metal soaps—i.e., calcium stearate and lithium stearate—on the formation of fibers in, and consequently the transparency of, a PP product obtained by injection molding. As is well known, calcium stearate is often added to PP as an acid neutralizer.

## 2. Materials and Methods

### 2.1. Materials

A commercially available isotactic propylene homopolymer (PP, PM900A; SunAllomer Ltd., Tokyo, Japan) was used. Because it was provided in the powder form, no additive was mixed. Its melting point, measured by a differential scanning calorimeter, is 163 °C at a heating rate of 10 °C/min. The melt flow rate measured following JIS K7210 is 30 g/10 min at 230 °C under 2.16 kgf. The number- and weight-average molecular weights, measured by size exclusion chromatography, are 35,000 and 179,000, respectively. Tris(2,4-di-tert-butylphenyl)phosphite (Irgafos^®^ 168; BASF SE., Ludwigshafen, Germany) and pentaerythritol tetrakis(3-(3,5-di-tert-butyl-4-hydroxyphenyl)propionate) (Irganox^®^1010; BASF SE., Ludwigshafen, Germany) were used as thermal stabilizers. The content of each was 0.05 wt. %. Either calcium stearate (StCa; Nitto Kasei Kogyo K.K., Kanagawa, Japan) or lithium stearate (StLi; Nitto Kasei Kogyo K.K., Kanagawa, Japan) was used as an acid neutralizer. The content of each was 0.05 wt. %. 1,3:2,4-Bis-*o*-(4-methylbenzylidene)-d-sorbitol (MDBS; GEL ALL^®^ MD; New Japan Chemical Co. Ltd., Osaka, Japan) was used as the sorbitol-based crystal nucleating agent. The contents were 0.1, 0.2, and 1.0 wt. %. The melting point of MDBS is 262 °C.

The article "Effect of Neutralizer on Transparency of Nucleating Agent-Containing Polypropylene" was published in 2021. Journal: Polymers (Basel).

### 2.2. Sample Preparation

PP, MDBS, the thermal stabilizers, and one of the acid neutralizers were mixed at 240 °C. According to a previous study [25], 1 wt. % of MDBS is fully dissolved in molten PP at this temperature. A corotating twin-screw extruder (KZW15TW-45MG-NH; Technovel Corp., Osaka, Japan) having kneading zones was used as a mixing device. The length-to-diameter ratio was 45 with a screw diameter of 15 mm. The screw rotational speed was 250 rpm, and the output rate was controlled at 3.6 kg/h by using a weighing feeder. The temperature profile of the extruder was as follows: C1/180 °C, C2/200 °C; C3/240 °C, C4/240 °C, adapter/240 °C, and die/240 °C. The strand was extruded through a circular die with a diameter of 5 mm, immediately cooled in a water bath at 25 °C, and cut into small pellets using a strand cutter. A sample without MDBS but with 0.05 wt. % StCa was also prepared as a reference.

The obtained pellets were molded into flat plates using an injection molding machine (PS40E5ASE; Nissei Plastic Industrial Co., Ltd., Nagano, Japan) with a clamping capacity of 40 tons. The dimension of the plates was as follows; 35 mm in width, 40 mm in length, and 0.5–3.0 mm in thickness. The injection-molding was carried out at the following conditions; temperature profile of the barrel (C1/180 °C, C2/190 °C, C3/195 °C, and C4/200 °C); injection-pressure 11.7 MPa; holding pressure 1.4 MPa; injection-time 10 s (for the plates with 0.5 and 1.0 mm thicknesses) and 15 s (for those with 2.0 and 3.0 mm thicknesses); cooling time 10 s; and screw rotation speed 100 rpm. The mold temperature was controlled at 40 °C.

## 3. Measurements

The optical transparency of each specimen was evaluated at room temperature using a direct reading haze meter (Toyo Seiki Seisaku-sho, Ltd., Tokyo, Japan). Haze is defined as the percentage of light transmitted through a specimen that is at least 2.5° away from the incident light due to forward scattering, and is the ratio of the intensity of diffuse transmission to that of total light transmission. Therefore, a specimen with good transparency has a low haze value. The measurements were performed five times for each sample, and the average value was calculated.

The temperature dependence of the dynamic tensile modulus of each sample was measured from −100 to 165 °C using a dynamic mechanical analyzer (Rheogel-E4000-DVE; UBM Co., Ltd., Kyoto, Japan). The frequency was 10 Hz, and the heating rate was 2 °C/min. Rectangular specimens (5 mm wide and 20 mm long) were cut from the 0.5-mm thick injection-molded plate. As shown in Figure 1, two types of specimens were prepared to investigate the mechanical anisotropy: one type with the long dimension parallel to the flow direction (the MD sample), and the other type with the long dimension perpendicular to the flow direction (the TD sample). Therefore, the direction of applied oscillatory strain coincided with the flow direction of the MD sample.

The article "Effect of Neutralizer on Transparency of Nucleating Agent-Containing Polypropylene" was published in 2021. Journal: Polymers (Basel).

Birefringence measurements were performed using a polarizing optical microscope (DMLP; Leica Microsystems GmbH, Wetzlar, Germany) with a compensator (Compensator B; Leica Microsystems GmbH, Wetzlar, Germany). As shown in Figure 2, a 2.5-μm thick sample was cut from a 0.5-mm thick injection-molded plate at −100 °C using an ultramicrotome equipped with a diamond knife (FCS; Leica Microsystems GmbH, Wetzlar, Germany).

The thermal analyses were performed in a nitrogen atmosphere using a differential scanning calorimeter (DSC 820; Mettler-Toledo International Inc., Greifensee, Switzerland). A 6-mg sample was placed in an aluminum pan, heated to 230 °C, and held at that temperature for 3 min to completely melt the PP. The sample was then cooled at a rate of 10 °C/min to determine the crystallization temperature.

The steady-state shear viscosity was measured at 180 °C using a capillary rheometer (140 SAS-2002; Yasuda Seiki Co., Ltd., Hyogo, Japan). A circular die that was 10 mm long, 1.0 mm in diameter, and had an entrance angle of 2π was used. Neither Bagley nor Rabinowitsch corrections were performed, because the viscosity was low.

The frequency dependency of the oscillatory shear modulus of each sample was determined using a cone-and-plate rheometer (MR-500; UBM Co., Ltd., Kyoto, Japan) at 180, 200, 210, and 220 °C in a nitrogen atmosphere. The diameter of the cone was 20 mm, and the cone angle was 4°.

Wide-angle X-ray diffraction (WAXD) patterns were obtained from a 0.5-mm thick injection-molded plate using an X-ray diffractometer (RINT2500; Rigaku Corp., Tokyo, Japan). The sample specimens were exposed for 15 min to a graphite-monochromatized Cu Kα radiation beam generated at 100 mA and 40 kV.

## 4. Results and Discussion

The steady-state shear viscosity under a pressure-driven capillary flow (Figure 3) was measured at 180 °C to evaluate the effect of a neutralizer, i.e., StCa or StLi. The content of MDBS was 1.0 wt. %. Shear viscosity $\eta_{a}$ and shear rate ${\overset{\cdot }{\gamma }}_{a}$ are the apparent values on the wall. In the experimental shear rate region, no flow instability, including shark-skin failure [42], was detected in either sample.

Neutralizers—i.e., metal soaps—sometimes act as lubricants, and thus induce wall slippage [43]. In the present study, however, the viscosity values of both samples were almost the same, indicating that the wall slippage was negligible. Considering the low content of the neutralizers—i.e., 0.05 wt. %—this is a reasonable result.

The article "Effect of Neutralizer on Transparency of Nucleating Agent-Containing Polypropylene" was published in 2021. Journal: Polymers (Basel).

Figure 4 shows plots of the haze values (with error bars) of the injection-molded plates versus thickness. Because the experimental error was quite small, the error bars were almost hidden by the symbols.

Figure 4 confirmed that the haze value decreases dramatically with the MDBS content. In particular, the thin plates are highly transparent. This can be attributed to a large correlation length in the skin layer due to the high degree of molecular orientation, and reduced light scattering from spherulites in the core. The figure also demonstrated that the identity of the neutralizer has a marked effect on the transparency, which was obvious at a low concentration of MDBS, i.e., 0.1 wt. %. The plates containing StLi had greater transparency (lower haze values) irrespective of the thickness. In the plates containing 1.0 wt. % of MDBS, the haze values followed the opposite order, i.e., the haze values of the plates with StCa were lower than those with StLi. Furthermore, when the MDBS content was 0.2 wt. %, there was almost no difference in the haze values, irrespective of the plate thickness.

The crystalline structure was evaluated from the WAXD profiles, as shown in Figure 5. Although it has been reported that StCa accelerates β-trigonal-form crystals, the diffraction peak ascribed to β-form crystals, denoted by the arrows in the figure, was weak for all the plates. The WAXD profiles also demonstrated that the crystallinity is greatly enhanced by MDBS.

Molecular orientation in the injection-molded plates was evaluated by birefringence. Figure 6 shows the birefringence distribution in the thickness direction. Because a 0.5-mm thick injection-molded plate was used, the position at 0.25 mm is the center of the plate. When spherulite texture was detected, the birefringence was plotted as zero.

MDBS greatly enhances the molecular orientation in the skin layer. Considering that the intrinsic birefringence of PP is approximately 4 × 10^−2^ [44,45,46], the plates containing MDBS had high orientation function values; the orientation function is the ratio of the measured birefringence to the intrinsic birefringence. Even in the core layer, in the absence of spherulite texture, there was some degree of orientation when MDBS was added. Therefore, MDBS was responsible for the high transparency. The level of molecular orientation was pronounced when the MDBS content was high, i.e., 1.0 wt. %. According to these measurements, there was no difference in orientation between the plates containing StLi and those containing StCa.

The article "Effect of Neutralizer on Transparency of Nucleating Agent-Containing Polypropylene" was published in 2021. Journal: Polymers (Basel).

The anisotropy in the dynamic mechanical properties was measured to evaluate the degree of molecular orientation. The tensile storage modulus (*E′*) of an MD sample is higher at low temperatures and lower at high temperatures than that of a TD sample [29,47,48]. This crossover behavior of *E*′ between the MD and TD samples was pronounced when the molecular orientation was high. As shown in Figure 7, the crossover behavior followed the following order: MDBS (1%)/StCa, MDBS (1%)/StLi, MDBS (0.1%)/StLi, MDBS (0.1%)/StCa, and PP without MDBS. This was the same order as for transparency.

Figure 8 shows the temperature dependence of the tensile loss modulus (*E*′′) of each MD sample. The peak area of the β dispersion ascribed to the glass-to-rubber transition was reduced by the addition of MDBS owing to the decrease in the amorphous region. Correspondingly, the α dispersion located between 50 and 130 °C, which is a mechanical relaxation associated with crystal grain boundaries, was enhanced by MDBS. When the MDBS content was 1.0 wt. %, the plate containing StCa produced a pronounced peak compared with that containing StLi. In contrast, when the MDBS content was 0.1 wt. %, the plate containing StLi produced a pronounced peak compared with that containing StCa. Therefore, StLi effectively enhances the nucleating activity of MDBS when the MDBS content is 0.1 wt. %.

Figure 9 shows the DSC cooling curves. A clear exothermic peak was detected in all the samples. The crystallization temperatures of the samples containing MDBS were higher than the crystallization temperature of pure PP. It should be noted that the crystallization temperature of the samples containing 0.1 wt. % of MDBS was greatly affected by the identity of the neutralizer. This indicated that the segregation/crystallization of MDBS occurred earlier in the sample containing StLi than in the sample containing StCa. The prompt formation of MDBS fibers is responsible for the reduced light scattering, i.e., low haze values. In contrast, when the content of MDBS was 1 wt. %, the sample containing StCa had a slightly higher crystallization temperature with a narrow peak than the sample containing StLi.

The network structure of the MDBS fibers in the molten PP was determined by evaluating the viscoelastic properties of the injection-molded plates. Figure 10 shows the angular frequency dependence of the shear storage modulus (*G*′) and the loss modulus (*G*′′) at 180 °C. The values for pure PP are denoted by the lines, which reveal the typical behavior of a simple polymer melt in the rheological terminal region. When the MDBS content was 1.0 wt. %, the *G*′ values formed a clear plateau in the low frequency region for both samples, which can be attributed to the network structure of MDBS fibers [14,49]. The plateau modulus of the sample containing StCa was higher than that of the sample containing StLi. This result demonstrated again that the segregation/crystallization of MDBS in molten PP was affected by the presence of a neutralizer, i.e., a well-developed network structure formed in the sample containing StCa when the MDBS content was 1.0 wt. %.

The article "Effect of Neutralizer on Transparency of Nucleating Agent-Containing Polypropylene" was published in 2021. Journal: Polymers (Basel).

The viscoelastic properties of the samples with 0.1 wt. % of MDBS appear to be similar to those of pure PP, irrespective of the identity of the neutralizer. However, the *G*′ values in the low frequency region of the samples containing MDBS were slightly higher than those of pure PP. This phenomenon was more obvious in the sample containing StLi, indicating that the impact of the neutralizer on the segregation/crystallization behavior of MDBS is dependent on the identity of the neutralizer as well as the MDBS content.

Figure 11 shows the master curves of *G*′ and *G*′′ for the samples containing 1.0 wt. % of MDBS. The reference temperature was 180 °C. The curves were shifted horizontally to superimpose the values in the high frequency region. Both systems had the same shift factor, confirming that the neutralizer does not affect the flow activation energy, which was approximately 40 kJ/mol—i.e., a typical value for PP [50,51].

Both moduli increased in the low frequency region at low temperatures, suggesting that the MDBS had segregated/crystallized and consequently had formed a network structure. The figure also demonstrates that the identity of the neutralizer affects these phenomena. The plateau values of *G*′ for the samples containing StCa were higher than those containing StLi in the temperature region at/below 210 °C when the MDBS content was 1.0 wt. %.

The viscoelastic properties and DSC cooling curves suggested that StLi effectively accelerates the segregation/crystallization of MDBS when the content is 0.1 wt. %. In contrast, when the MDBS content is 1.0 wt. %, StCa is more effective. These results correspond with the mechanical anisotropy evaluated by the dynamic tensile modulus, and with the transparency. Although the detailed mechanism is still unknown, one possible reason is as follows: StLi always accelerates the segregation/crystallization of MDBS, and StCa always delays the segregation/crystallization of MDBS. Consequently, MDBS agglomeration—not MDBS nanofiber formation—tends to occur readily when the MDBS content is high. The agglomerations are large enough to scatter visible light and thus result in the poor transparency as well as poor nucleating activity in PP. In the case of the sample containing a small amount of MDBS, the agglomeration barely occurs even with StLi. As a result, the sample containing StLi is transparent compared with that with StCa.

The article "Effect of Neutralizer on Transparency of Nucleating Agent-Containing Polypropylene" was published in 2021. Journal: Polymers (Basel).

Both StCa and sodium stearate are used as nucleating agents for poly(ethylene terephthalate) (PET) [52]. In this system, the cations in such nucleating agents interact with the ester bonds in PET, and become nucleating sites. Although MDBS does not have any ester bonds, it contains oxygen atoms, including those in its hydroxyl groups. Therefore, it is able to interact with metal stearates. In fact, sorbitol derivatives act synergistically with polar compounds to form network structures [40,41]. Moreover, the interaction between hydroxyl groups and lithium cations is known to be strong [53,54,55,56].

The following conclusions can be drawn from the obtained results. When the MDBS content is low, the segregation/crystallization of MDBS occurs early and enhances PP crystallization. StLi is preferably used for this purpose because it acts synergistically to form MDBS fibers. However, when the MDBS content is high, StCa works more effectively to form MDBS fibers. In the sample containing StLi, MDBS may have agglomerated when present in large amounts, especially in the core layer. This increases light scattering. Consequently, the transparency of the sample containing StLi is not as high as that of the sample containing StCa.

## 5. Conclusions

The effect of the neutralizer on the transparency of injection-molded PP plates containing MDBS was investigated. The addition of StLi instead of StCa—which is the conventional neutralizer—improved the transparency of a plate when the amount of MDBS was low. The prompt formation of MDBS fibers through segregation/crystallization induced by the addition of StLi is responsible for the phenomenon. However, as the amount of MDBS increased, the advantage of StLi was lost, and the plate containing StCa exhibited better transparency. The molecular orientation of the injection-molded plates was characterized by the anisotropy in the dynamic tensile modulus. This suggested that transparency is enhanced by an increase in molecular orientation. Furthermore, the PP crystallization behavior and the formation of an MDBS network in the molten PP corresponded well with the transparency.

## Figures and Tables

**Figure 1:** Sample specimens for dynamic mechanical analysis.

**Figure 2:** Samples for birefringence measurements.

**Figure 3:** Flow curves at 180 °C for the samples with calcium stearate (StCa; circles) and lithium stearate (StLi; diamonds).

The article "Effect of Neutralizer on Transparency of Nucleating Agent-Containing Polypropylene" was published in 2021. Journal: Polymers (Basel).

**Figure 4:** Haze values of the injection-molded plates with calcium stearate (StCa; open symbols) and lithium stearate (StLi; closed symbols). The 1,3:2,4-bis-*o*-(4-methylbenzylidene)-d-sorbitol (MDBS) contents were: 1.0 wt. % (**circles**), 0.2 wt. % (**diamonds**), 0.1 wt. % (**triangles**), and 0 wt. % (**squares**).

**Figure 5:** Wide-angle X-ray diffraction (WAXD) patterns of the plates with (**a**) calcium stearate (StCa) and (**b**) lithium stearate (StLi).

**Figure 6:** Distribution of birefringence in the thickness direction of the plates with calcium stearate (StCa; open symbols) and lithium stearate (StLi; closed symbols). The 1,3:2,4-bis-*o*-(4-methylbenzylidene)-d-sorbitol (MDBS) contents were: 1.0 wt. % (**circles**), 0.1 wt. % (**triangles**), and 0 wt. % (**squares**).

**Figure 7:** Temperature dependence of the tensile storage modulus (*E*′) of the 0.5-mm thick plates. Closed symbols: MD samples (prepared with the long dimension parallel to the flow direction); and open symbols: TD samples (prepared with the long dimension perpendicular to the flow direction).

**Figure 8:** Temperature dependence of the tensile loss modulus (*E*′′) of the 0.5-mm thick plates (MD samples—i.e., prepared with the long dimension parallel to the flow direction); calcium stearate (StCa; open symbols) and lithium stearate (StLi; closed symbols). The MDBS contents were: 1.0 wt. % (**circles**), 0.1 wt. % (**triangles**), and 0 wt. % (**squares**).

**Figure 9:** Differential scanning calorimeter (DSC) cooling curves of isotactic polypropylene (PP) and PP/MDBS. PP = isotactic polypropylene; MDBS = 1,3:2,4-bis-*o*-(4-methylbenzylidene)-d-sorbitol.

**Figure 10:** Frequency dependence of the shear storage modulus (*G*′; closed symbols and solid line) and the loss modulus (*G*′′; open symbols and dotted line) at 180 °C for the samples containing (**left**) 1.0 wt. % and (**right**) 0.1 wt. % of 1,3:2,4-bis-*o*-(4-methylbenzylidene)-d-sorbitol (MDBS). Calcium stearate (StCa; **circles**) and lithium stearate (StLi; **diamonds**). The lines represent the data for pure PP.

**Figure 11:** Master curves of the oscillatory shear moduli (**left**) *G*′ and (**right**) *G*′′ for the samples containing calcium stearate (StCa; **top**) and lithium stearate (StLi; **bottom**) at the reference temperature of 180 °C. The 1,3:2,4-bis-*o*-(4-methylbenzylidene)-d-sorbitol (MDBS) content was 1.0 wt. %. **Circles**: 180 °C; **diamonds**: 200 °C; **triangles**: 210 °C; and **squares**: 220 °C.

## Data Availability

The data presented in this study are available on request from the corresponding author.
